The article "Increased breast tissue receptor activator of nuclear factor-κB ligand (RANKL) gene expression is associated with higher mammographic density in premenopausal women" was published in 2017. Journal: Oncotarget.

# Increased breast tissue receptor activator of nuclear factor-κB ligand (RANKL) gene expression is associated with higher mammographic density in premenopausal women

**DOI:** 10.18632/oncotarget.17909

**Published:** 2017-05-17

**Authors:** Adetunji T. Toriola, Ha X. Dang, Ian S. Hagemann, Catherine M. Appleton, Graham A. Colditz, Jingqin Luo, Christopher A. Maher

**Affiliations:** ^1^ Department of Surgery, Division of Public Health Sciences, and Siteman Cancer Center, Washington University School of Medicine, St. Louis, MO, USA; ^2^ The McDonnell Genome Institute, and Department of Medicine, Washington University, St. Louis, MO, USA; ^3^ Genomics and Pathology Services, Department of Pathology and Immunology, Washington University School of Medicine, St. Louis, MO, USA; ^4^ Division of Diagnostic Radiology, Department of Radiology, Washington University School of Medicine, St. Louis, MO, USA

**Keywords:** mammographic density, breast cancer, RANKL, premenopausal women, prevention

## Abstract

Increased mammographic breast density is associated with a 4–6-fold increased risk of breast cancer, yet lifestyle factors that can reduce dense breasts are yet to be identified, and viable prevention strategies to reduce breast density-associated breast cancer development are yet to be developed. We investigated the associations of breast tissue receptor activator of nuclear factor-κB (RANK) pathway gene expression with mammographic density in 48 premenopausal women, with no previous history of cancer. Gene expression levels were measured in total RNA isolated from formalin-fixed paraffin-embedded breast tissue samples, using the NanoString nCounter platform. Mammographic density was classified based on the American College of Radiology Breast Imaging Reporting and Data (BI-RADS). Linear regression was used to evaluate associations between gene expression and mammographic density. The mean age of participants was 44.4 years. Women with higher breast tissue RANKL (*TNFSF11*) (*p*-value = 0.0076), and TNF (*p*-value = 0.007) gene expression had higher mammographic density. Our finding provides mechanistic support for a breast cancer chemoprevention trial with a RANKL inhibitor among high-risk premenopausal women with dense breasts.

## INTRODUCTION

Increased mammographic breast density is associated with a 4–6-fold increased risk of breast cancer [1–3]. Each 1% increase in percent mammographic density is associated with a 3% increase in breast cancer risk among women using estrogen plus progestin [1]. Estimates of attributable risk suggest that having dense breasts may account for 28–33% of breast cancer cases [4]. Furthermore, 2.4 million premenopausal women in the United States have extremely dense breasts [5]. Hence, providing targeted prevention to these women could have a major impact on reducing breast cancer incidence. Nevertheless, lifestyle factors that can reduce dense breasts are yet to be identified, and viable prevention strategies to reduce mammographic breast density-associated breast cancer development are yet to be developed.

The article "Increased breast tissue receptor activator of nuclear factor-κB ligand (RANKL) gene expression is associated with higher mammographic density in premenopausal women" was published in 2017. Journal: Oncotarget.

Preclinical studies demonstrating important functional roles for the receptor activator of nuclear factor-κB (RANK) pathway, a member of the tumor necrosis factor (TNF) superfamily in breast development suggest that targeting this pathway could have utility in primary breast cancer prevention. RANK is the signaling receptor for RANK ligand (RANKL), while osteoprotegerin (OPG) acts as a soluble decoy receptor [6]. RANKL is required for mammary epithelial cell proliferation [7], an essential part of breast density. Seminal experimental studies revealed that RANKL signaling mediates the major proliferative response of mammary epithelium to progesterone, and progesterone-driven expansion of mammary stem cells [8, 9]. Progesterone is a breast mitogen; it increases breast density, and is a risk factor for breast cancer, independent of estrogen [10, 11]. Notably, disruption of RANKL signaling attenuates progestin-driven mammary epithelial cell proliferation, and reduces the onset of mammary tumors in experimental studies [7, 8, 12]. In addition, novel data show that RANKL signaling could be important in BRCA1 mutation-driven mammary cancer [13], and RANKL inhibition in breast organoids derived from pre-neoplastic BRCA mutation tissue attenuated progesterone-induced proliferation [13, 14]. Therefore, targeting RANKL signaling could present a path to reducing mammographic breast density, as well as breast-density associated breast cancer development. However, to the best of our knowledge, no study has evaluated how RANKL signaling influences mammographic density. Here, we investigated for the first time the associations of breast tissue *RANK* pathway gene expression with mammographic density in premenopausal women.

## RESULTS

The mean age of women in our study was 44.4 years (Table 1). The mean body mass index (BMI) was 27.5 kg/m^2^. In line with the mammographic density distribution among US women, the majority of women (N=20, 41.7%) in our study had heterogeneously dense breasts, 18 (37.5%) had scattered areas of fibroglandular density and 9 (18.8%) had extremely dense breasts. We observed statistically significant associations between breast tissue *RANKL* (*TNFSF11*) and *TNF* gene expression and mammographic density, but no statistically significant associations between breast tissue expression of other genes (e.g. *CYP27A1, EGFR, ESR1, IGF-1, IGFBP-3, IL-6*) and mammographic density (Figure 1A). Women with higher breast tissue *RANKL* (*TNFSF11*) (*p*-value=0.0076), and *TNF* (*p*-value = 0.007) gene expression had higher mammographic density (Figure 1B and 1C). Findings were similar in sensitivity analyses (*P*-value for *RANKL* gene expression was 0.012) where we re-categorized the women into lower mammographic density and higher mammographic density.

The article "Increased breast tissue receptor activator of nuclear factor-κB ligand (RANKL) gene expression is associated with higher mammographic density in premenopausal women" was published in 2017. Journal: Oncotarget.

**Table 1:** Characteristics of 48 premenopausal women from the St. louis breast tissue registry who provided breast tissue and mammographic density data

	Mean (Standard deviation)
**Age, years**	44.38 (4.0)
**Body Mass Index, kg/m^2^**	27.45 (5.9)
	**Number of observations (%)**
**Race**	
White Non-Hispanic	33 (68.8)
African American	12 (25.0)
Others	3 (6.2)
**Mammographic density**	
1	1 (2.1)
2	18 (37.5)
3	20 (41.7)
4	9 (18.8)

**Figure 1:** Breast tissue TNFSF11 (RANKL) and TNF gene expression and mammographic density in premenopausal women Volcano plot showing that breast tissue *TNFSF11* (RANKL) and *TNF* gene expression are associated with mammographic density in premenopausal women, but not gene expression of other proteins (e.g. *IGF1*, *EGFR*) (**A**) Figures showing that higher breast tissue *RANKL* (*TNFSF11*, *p*-value = 0.0076) and TNF (*p*-value = 0.0069) gene expression are associated with higher mammographic density in premenopausal women (**B** and **C**).

## DISCUSSION

We provide the first evidence showing that *RANKL* gene expression is associated with mammographic density in premenopausal women. Our finding has translational potentials, and provides additional context on targeting RANKL signaling in breast cancer prevention. Recent data showing that RANKL signaling may drive BRCA1 mutation driven mammary cancer has generated interest in targeting RANKL inhibition for chemoprevention in women with BRCA1 mutation. A dense breast on mammogram confers similar magnitude of risk (i.e. 4–6 fold) as BRCA1 mutation [15]. Importantly, breast cancer risk decreases among women whose mammographic density decreased over time compared to women whose density stayed the same [16]. Therefore, RANKL inhibition with denosumab could be a viable breast cancer prevention strategy in high-risk premenopausal women [17] with dense breasts.

RANKL signaling regulates the development of the lobulo-alveolar mammary structures during pregnancy and the formation of lactating mammary glands [18–20]. RANK overexpression in the mammary epithelia impairs alveolar differentiation and lactation [21]. RANK and RANKL knock out mice display a complete defect in the formation of lactating mammary glands, due to decreased proliferation and survival of mammary epithelial cell, similar to that observed in progesterone receptor B knockout mice [18, 22, 23]. RANKL signaling also activates downstream signaling cascades such as NF-kB and cyclin D1 [6, 12], which are key pathways, involved in breast cancer development [6, 12]. Very recent studies conducted in Europe demonstrated that elevated serum RANKL levels are associated with increased breast cancer risk among women with high progesterone levels [24], while another study reported that elevated OPG levels are associated with increased breast cancer risk [25]. Our study adds to findings from these initial studies indicating that the RANK pathway plays an important role in breast cancer development.

The article "Increased breast tissue receptor activator of nuclear factor-κB ligand (RANKL) gene expression is associated with higher mammographic density in premenopausal women" was published in 2017. Journal: Oncotarget.

Besides being a strong risk factor for breast cancer, mammographic density and breast cancer share similar biological and genetic pathways [26, 27]. Thus, being a strong intermediate phenotype for breast cancer provides additional support for targeting women with dense breasts in breast cancer chemoprevention. Mammographic density is highly heritable, with suggestion that genetic factors may explain 60% of the variance [28]. Nevertheless, the loci identified to date explain < 3% of the variance in mammographic density [27, 29] indicating that many genetic determinants are yet to be identified. Although some known breast cancer susceptibility loci are also associated with mammographic density [27], mutations in highly penetrant breast cancer genes; BRCA1 and BRCA 2 genes have not been found to be associated with mammographic density [30].

Aside from reproductive factors and alcohol consumption, most of the other lifestyle factors that can be modified to reduce breast cancer risk (e.g. obesity, menopausal hormone use) are only relevant to disease among postmenopausal women. Likewise, adult diet is not related to mammographic density [31], hence, dietary and lifestyle modifications are not likely to impact mammographic density. Tamoxifen is the only approved chemoprevention agent in premenopausal women, but uptake is very low due to risk of serious side effects [32, 33]. Therefore, denosumab could be a more attractive chemoprevention option in high-risk premenopausal women because of its safety profile [34]. It is currently in clinical use for the management of osteoporosis and for preventing bone loss, as well as fractures associated with cancer therapies and bone metastases [34], whereas tamoxifen negatively impacts bone health in premenopausal women [35]. Further, unlike tamoxifen, which must be taken daily, denosumab is typically given every six months [34]. Hence, chemoprevention with denosumab might require administration every 6 months, which should considerably help improve compliance.

The article "Increased breast tissue receptor activator of nuclear factor-κB ligand (RANKL) gene expression is associated with higher mammographic density in premenopausal women" was published in 2017. Journal: Oncotarget.

In conclusion, findings from our study provide essential mechanistic support for targeting RANKL signaling in reducing breast cancer development in high-risk premenopausal women with dense breasts.

## MATERIALS AND METHODS

### Study population

We identified 48 premenopausal women, with no previous history of cancer, who had a screening mammogram and subsequent breast biopsy at the Joanne Knight Breast Health Center, Washington University School of Medicine (WUSM), St. Louis, MO between December 2008 and 2015, and afterwards had their breast tissue samples stored in the well-annotated St. Louis Breast Tissue Registry (SLBTR), Department of Surgery, WUSM. The SLBTR was created in 1993 as part of the National Cancer Institute (NCI) Cooperative Breast Cancer Tissue Resource. It maintains a publicly available supply of archival breast tissue specimens coupled with clinical, pathological, and follow-up data from five hospitals in the St. Louis region. Breast tissue specimens were evaluated for pathologic diagnosis by breast pathologists using standard diagnostic criteria. Eligibility criteria for our study included (i) women must be premenopausal at the time of mammogram; (ii) no history of ovariectomy (ii) no evidence of cancer on breast biopsy, (iii) breast biopsy must have been done within 30 days of having a mammogram. Exclusion criteria were (i) history of any cancer, (ii) selective estrogen receptor modulator, aromatase inhibitors, or bisphosphonates use within 6 months of having a mammogram, (iii) history of breast implants, reduction mammoplasty, or augmentation.

### RANK pathway gene expression

Gene expression levels were measured in total RNA isolated from formalin-fixed paraffin-embedded (FFPE) breast tissue samples, using the NanoString nCounter platform. We selected this platform because it reliably monitors gene expression in archival specimens, has technical reproducibility, and allows direct measurement of RNA expression levels without enzymatic reactions or bias. In addition to *RANKL* gene, we also targeted known genes in TNF superfamily such as *TNF* and *TNFRSF13B*. We designed nanoString probes to monitor gene expression of additional genes (such as *CYP27A1, EGFR, ESR1, IGF-1, IGFBP-3, IL-6*) that may be related to breast cancer risk. Gene expression was performed at the McDonnell Genome Institute (MGI), WUSM. Digital transcript counts from the NanoString nCounter assay was normalized using the housekeeping genes (*ACTB, RPLP0,* and *SF3A1*) following the manufacturer’s guidelines.

### Mammographic density assessment

Mammographic density was classified based on the American College of Radiology Breast Imaging Reporting and Data (BI-RADS) system as (i) Almost entirely fatty, (ii) Scattered areas of fibroglandular density, (iii) Heterogeneously dense, (iv) Extremely dense. In sensitivity analyses, we categorized the women into 2 groups; lower mammographic density group (entirely fatty breast and scattered areas of fibroglandular patterns), and higher mammographic density group (heterogeneously dense and extremely dense).

The article "Increased breast tissue receptor activator of nuclear factor-κB ligand (RANKL) gene expression is associated with higher mammographic density in premenopausal women" was published in 2017. Journal: Oncotarget.

### Statistical analyses

NanoString nCounter transcript counts were normalized to the positive spike-in control probes, and subsequently to the housekeeping genes (*ACTB, RPLP0*, and *SF3A1*). Background was measured by negative spike-in controls. For each sample, a geometric mean of the counts of housekeeping genes was calculated. The average of the housekeeping geometric means across samples was also calculated and then divided by each sample’s housekeeping genes’ geometric mean to obtain the scaling factor for the corresponding sample. A gene was considered to be expressed if its normalized count was higher than the mean normalized count of the negative control probes in at least 10 samples. Normalized counts were log transformed prior to downstream analysis. A linear regression was used to evaluate associations between gene expression and mammographic density. All analyses and visualizations were performed in R software version 3.1.2.
